This article has been retracted.

# Treatment comparison of femoral shaft with femoral neck fracture: a meta-analysis

**DOI:** 10.1186/s13018-019-1496-z

**Published:** 2020-01-20

**Authors:** Yao Lu, Yakang Wang, Zhe Song, Qian Wang, Liang Sun, Cheng Ren, Hanzhong Xue, Zhong Li, Kun Zhang, Dingjun Hao, Yang Zhao, Teng Ma

**Affiliations:** Department of Orthopaedic Surgery, HongHui Hospital, Xi’an Jiaotong University, Xi’an, 710054 Shaan’xi Province China

**Keywords:** Reconstruction nail, Hollow screw, Plate, Femoral shaft with femoral neck fracture

## Abstract

**Background:**

To compare the efficacy and complications between reconstruction nail and hollow screw+plate in patients with femoral shaft and femoral neck fracture.

**Methods:**

The full text of studies on clinical efficacy involving reconstruction nail and hollow screw+plate was retrieved from multiple databases. Review Manager 5.0 was adopted for meta-analysis, sensitivity analysis, and bias analysis. The meta-analysis was conducted with respect to the operation time, blood loss, healing time of the femoral shaft, healing time of the femoral neck, and complications. Finally, 10 studies met the eligibility criteria, including 991 patients.

**Results:**

The meta-analysis suggested better characteristics for the reconstruction nail compared with the hollow screw+plate regarding operation time (OR = − 82.41, 95% CI [− 91.72, − 73.10], *P* < 0.00001; *P* for heterogeneity < 0.00001, *I*^*2*^ = 98%), blood loss (OR = − 388.01, 95% CI [− 422.95, − 353.06], *P* < 0.00001; *P* for heterogeneity < 0.00001, *I*^*2*^ = 99%), healing time of femoral shaft (MD = − 3.89, 95% CI [− 4.74, − 3.05], *P* < 0.00001; *P* for heterogeneity < 0.00001, *I*^*2*^ = 99%), healing time of femoral neck (MD = − 4.04, 95% CI [− 4.33, − 3.75], *P* < 0.00001; *P* for heterogeneity = 0.008, *I*^*2*^ = 60%), and complications (OR = 0.47, 95% CI [0.31, 0.73], *P* = 0.0006; *P* for heterogeneity = 1.00, *I*^*2*^ = 0%).

**Conclusion:**

This meta-analysis shows that a reconstruction nail is a more efficient and safer treatment than a hollow screw+plate for patients with femoral shaft and femoral neck fracture.

## Background

A femoral shaft combined with femoral neck fracture is a common condition. The incidence of this injury accounts for about 10% of the total incidence of femoral shaft fractures. The femoral shaft and femoral neck fracture are mostly caused by trauma [1–3]. When the hip is in the flexion abduction position, and the knee is in the flexion position, the assault from the front and the inertia of the body result in an axial force. If the femoral shaft fracture cannot absorb all the energy, the residual force is transmitted to the femoral neck, resulting in femoral neck fracture [4–6]. If the hip is in the adduction position when it is injured, the posterior dislocation of the hip often occurs in addition to the fracture of the femoral head.

Although the treatment of the femoral neck with femoral shaft fracture is difficult, several methods have been reported [7, 8]. In this study, the femoral reconstruction nail fixation, the plate system fixation, and the hollow nail fixation are discussed. Femoral reconstruction nail fixation has the following advantages: (a) fixation of the two fractures, axis fixation, and control of the length in multiple femoral shaft fractures and (b) closure of the pin, avoid damaging to local blood circulation, avoid peeling off the local periosteum, and minimal trauma. Meanwhile, the reconstruction nails have the following shortcomings: (a) great technical difficulty and the surgery should take into account both reduction and fixation, especially in the displacement of femoral neck fracture reduction and fixation operation and (b) femoral neck fractures can be shifted and rotated while placing a pin [9–11].

The advantages of the plate system in fixing the femoral shaft fracture and hollow nail in fixing the femoral neck fracture include simple operation, direct reduction, and control of the femoral shaft rotation. However, the disadvantages of large trauma, excessive bleeding, extensive peeling of periosteum, and high probability of nonunion were reported [12, 13]. The main complications of femoral shaft combined with femoral neck fracture include nonunion of the femoral neck fracture, femoral head necrosis, coxa varus deformity, nonunion of the femoral shaft fracture, and malunion [14].

Several articles have compared these two methods, encompassing various research designs, recruitment and exclusion criteria, and measurements. Currently, only a few meta-analyses have compared the reconstruction nail and hollow screw+plate. Therefore, a meta-analysis was conducted to evaluate the clinical efficacy and safety of these two methods comprehensively.

## Methods

### Search strategy

The comparison between reconstruction nail and hollow screw+plate was comprehensively analyzed. The references from January 2010 to October 2018 were searched from PubMed, Springer, Embase, Wiley-Blackwell, and Chinese Journal Full-text Database.

Two authors searched the articles independently using the following keywords: (1) reconstruction nail; (2) hollow screw; (3) femoral shaft; and (4) femoral neck. These search terms were assembled using “and” to search the database for the related articles. In order to obtain additional relevant studies with high accuracy, the reference list of each retrieved article was also reviewed.

### Citation selection

All articles after the first screening were further examined by two other researchers. The titles and abstracts of these articles were screened independently and stringently. If the study was relevant, the full-text article was obtained.

The following inclusion criteria were required to be fulfilled by the included studies:

1. A randomized control trial study or a controlled clinical trial study;
2. Comparison of the treatment between reconstruction nail and hollow screw+plate;
3. Availability of full-text.

Exclusion criteria:

1. Not a randomized study;
2. Studies on other treatments other than reconstruction nail or hollow screw+plate;
3. Studies are lacking outcome measures or comparable results.

Finally, two different researchers jointly identified the articles. Subsequently, whether the study fulfilled the above requirements or not was examined. In case of any discrepancy or disagreement, a third investigator was consulted for consensus.

### Search results

A preliminary search in the electronic database retrieved 362 related titles and abstracts. After a thorough review, 10 articles were found to fulfill all the inclusion criteria. The remaining 352 articles were excluded due to the following reasons: repeated, irrelevant studies, no control groups, incomplete data or comparisons, other operations, reviews, or incomplete articles. Figure 1 presents a schematic of the identification, inclusion, and exclusion criteria of the studies, thereby summarizing the search process and the reasons for exclusion.

**Fig. 1:** Schematic of the study identification and inclusion and exclusion criteria

### Data extraction

Two reviewers read the full text and extracted the relevant data from each study into Microsoft Excel. The characteristics extracted from each study included the first author’s name, publication year, year of onset, sample size (reconstruction nail/hollow screw+plate), the age range of patients, and outcome parameters with respect to the treatment of reconstruction nail and hollow screw+plate.

### Statistical analysis

Meta-analysis was performed by Revman 5.0 (Cochrane Collaboration, 2011) to assess the differences in the clinical efficacy between reconstruction nail and hollow screw+plate and to assess the publication bias. *I*^*2*^ statistics reflected the level of heterogeneity. When the heterogeneous *I*^*2*^ statistic was > 50%, a random-effects model was used to obtain moderate or high heterogeneity; otherwise, a fixed-effects model was utilized.

Quality evaluation was assessed by the risk of bias table in the software. Seven criteria were employed for the evaluation: random sequence generation, allocation concealment, blinding of participants and personnel, blinding of outcome assessment, incomplete outcome data, and selective reporting and other bias. In addition, a funnel plot was constructed to estimate the putative publication bias.

## Results

### Characteristics of the included studies

Table 1 lists the first author’s name, year of publication, age of onset, sample size (reconstruction nail/hollow screw+plate), age range of patients, and outcome parameters for each study. These articles were published from 2010 to 2018. The sample size was between 15 and 466. The studies encompassed 991 patients with femoral shaft and femoral neck fracture, including 487 in the reconstruction nail group and 504 in the hollow screw+plate group.

**Table 1:** Characteristic of the included studies

Study	Year	Language	Country	Age range (mean)	Groups	*n*	Years of onset
Akgul [15]	2016	English	Turkey	17.6 ± 1.8	Reconstruction nail	5	September 2007 to June 2013
					Hollow screw+plate	10	
Boese [16]	2016	English	Germany	18.2 ± 2.1	Reconstruction nail	8	October 2008 to June 2010
					Hollow screw+plate	9	
Genest [17]	2018	English	Germany	54.7 ± 12.1	Reconstruction nail	15	June 2010 to July 2016
					Hollow screw+plate	15	
Jiang [18]	2015	English	China	62.4 ± 18.7	Reconstruction nail	233	January 2009 to October 2014
					Hollow screw+plate	233	
Kovala k[19]	2017	English	Turkey	74.1 ± 4.1	Reconstruction nail	13	January 2009 to January 2015
					Hollow screw+plate	18	
Maranho [20]	2018	English	America	22.3 ± 1.7	Reconstruction nail	53	May 2000 to March 2014
					Hollow screw+plate	49	
Oh [21]	2017	English	Japan	78.2 ± 7	Reconstruction nail	10	August 2015 to February 2017
					Hollow screw+plate	11	
Ripamonti [22]	2014	English	Italy	68.4 ± 9.5	Reconstruction nail	38	April 2000 to March 2010
					Hollow screw+plate	166	
Sangeux [23]	2015	English	Australia	56.7 ± 2.3	Reconstruction nail	11	February 2002 to June 2010
					Hollow screw+plate	11	
Yamauchi [24]	2016	English	Japan	72.1 ± 11.2	Reconstruction nail	101	January 2010 to January 2012
					Hollow screw+plate	99	

### Quality assessment

The deviation table in the Review Manager 5.0 tutorial was used to assess the risk of each study by applying the criteria for evaluating the design-related deviations. The risk of bias in the present study is summarized in Figs. 2 and 3. The participants and respondents had a high risk of blindness due to significant differences between the reconstruction nail and hollow screw+plate groups.

**Fig. 2:** Assessment of the quality of the included studies: low risk of bias (green hexagons), unclear risk of bias (yellow hexagons), and high risk of bias (red hexagons)

**Fig. 3:** Quality assessment of included studies

### Results of meta-analysis

#### Meta-analysis on the operation time

A total of 10 studies were focused on the duration of the operation. Figure 4 illustrates the operation time of the reconstruction nail and hollow screw+plate groups. Moreover, statistically significant differences were observed in the operation time between reconstruction nail and hollow screw+plate. The current meta-analysis suggested a significant difference in the operation time between the reconstruction nail and hollow screw+plate (odds ratio (OR) = − 82.41, 95% confidence interval (CI): − 91.72 to − 73.10, *P* < 0.00001; *P* for heterogeneity < 0.00001, *I*^*2*^ = 98%). The operation time of the hollow screw+plate was higher than that of the reconstruction nail. When the data were categorized into two subgroups according to age, the *I*^2^ value changed from 98 to 24.7% (Fig. 5).

**Fig. 4:** Forest plot for operation time in reconstruction nail and hollow screw+plate groups

**Fig. 5:** Forest plot for subgroup analysis of operation time in reconstruction nail and hollow screw+plate groups

#### Meta-analysis on the blood loss

The forest plot for meta-analysis on blood loss is depicted in Fig. 6. The results demonstrated that the blood loss in the hollow screw+plate group was higher than that with reconstruction nail (OR = − 388.01, 95% CI: − 422.95 to − 353.06, *P* < 0.00001; *P* for heterogeneity < 0.00001, *I*^*2*^ = 99%). In the subgroup analysis of blood loss, the *I*^2^ value changed from 99 to 0% (Fig. 7).

**Fig. 6:** Forest plot for blood loss in reconstruction nail and hollow screw+plate groups

**Fig. 7:** Forest plot for subgroup analysis of blood loss in reconstruction nail and hollow screw+plate groups

#### Meta-analysis on the healing time of femoral shaft

The included studies on the healing time of the femoral shaft are shown in Fig. 8. The overall result indicated that the healing time of femoral shaft with hollow screw+plate was higher than that with reconstruction nail (MD = − 3.89, 95% CI: − 4.74 to − 3.05, *P* < 0.00001; *P* for heterogeneity < 0.00001, *I*^*2*^ = 99%. In the subgroup analysis for the healing time of the femoral shaft, the *I*^2^ value changed from 99 to 66.7% (Fig. 9).

**Fig. 8:** Forest plot for healing time of femoral shaft in reconstruction nail and hollow screw+plate groups

**Fig. 9:** Forest plot for subgroup analysis of healing time of femoral shaft in reconstruction nail and hollow screw+plate groups

#### Meta-analysis on the healing time of femoral neck

In the present meta-analysis, 10 studies were conducted on the comparison of the healing time of the femoral neck (Fig. 10). Statistically significant differences were detected between the reconstruction nail and hollow screw+plate, and the combined results showed that patients required more healing time for the femoral neck in hollow screw+plate as compared to the reconstruction nail (MD = − 4.04, 95% CI: − 4.33 to − 3.75, *P* < 0.00001; *P* for heterogeneity = 0.008, *I*^*2*^ = 60%).

**Fig. 10:** Forest plot for healing time of femoral neck in reconstruction nail and hollow screw+plate groups

#### Meta-analysis about complications

The articles addressing the complications of surgery were included. As shown in Fig. 11, significant difference in the complication between reconstruction nail and hollow screw+plate was observed, and the incidence with hollow screw+plate was higher than that with reconstruction nail (OR = 0.47, 95% CI: 0.31–0.73, *P* = 0.0006; *P* for heterogeneity = 1.00, *I*^*2*^ = 0%).

**Fig. 11:** Forest plot for complications in reconstruction nail and hollow screw+plate groups

### Sensitivity analysis

According to the meta-analysis, the heterogeneity of the operation time was high (*I*^2^ = 98%). As shown in Fig. 12, the low heterogeneity of the operation time might be attributed to the different results of each study. After excluding the study by Kovalak (2017), *I*^2^ was altered to 97%, which supported the robustness of this study.

**Fig. 12:** Forest plot for the sensitivity analysis in operation time between reconstruction nail and hollow screw+plate groups

### Bias analysis

Funnel plots of operation time with reconstruction nail and hollow screw+plate were constructed, including all the studies. The results showed moderate symmetry and little publication bias (Fig. 13). The result of Egger’s test did not provide any significant evidence of potential publication bias (*t* = 1.22, *P* = 0.267).

**Fig. 13:** Begg’s funnel plot of publication bias

## Discussion

A femoral shaft fracture combined with a femoral neck fracture is a relatively serious injury. In recent years, the literature reports an upward trend of the fracture [15]. The increase in the incidence of this combined fracture is attributed to the increased awareness of the fracture and the improvement of first aid ability to improve the patients’ life quality [15, 16]. A majority of the fracture is caused by trauma. Typically, indirect violence occurring along the femoral shaft causes hip flexion, abduction, and knee flexion.

In the case of femoral shaft fracture combined with femoral neck fracture, surgery is better than traction. Nonetheless, the reconstruction of the intramedullary nail is an optimal choice [17, 18]. The design of the femoral reconstruction intramedullary nail conforms to the physiological axis of the human femur and belongs to the central internal splint frame structure. Additionally, fretting at the fracture end during early movement or partial weight-bearing can promote callus growth.

The plate system femoral shaft fracture fixation with cannulated nail femoral neck fracture fixation presents the advantages of simple operation, direct reduction, and effectively reduces the incidence of femoral shaft rotation [19]. However, defects such as large surgical trauma, important bleeding, and high probability of non-union of plate fixation exist.

Currently, only limited studies have compared the reconstruction nail and hollow screw+plate for femoral shaft with femoral neck fracture. Moreover, the indicators and sample sizes were restricted. Furthermore, additional indicators and an increased sample size are needed for deeper study. In this study, the difference in the operation time and the healing time of the femoral shaft and femoral neck in the reconstruction nail and hollow screw+plate groups was significant. Thus, this phenomenon demonstrated that a reconstruction nail is a better treatment than a hollow screw+plate with respect to clinical efficacy. This result was similar to that by Song at el., which reported the reconstruction nail was deemed a more efficient therapy than a hollow screw+plate [18].

The comparison of blood loss and complications revealed that the value in the hollow screw+plate group was significantly higher than that in the reconstruction nail group. Watson and Moed stated that a reconstruction nail is a safer treatment than a hollow screw+plate, which is consistent with the current results [19].

All the results demonstrated that a reconstruction nail is better therapy than a hollow screw+plate in the treatment of patients with femoral shaft and femoral neck fracture. These results were coincident with those previous researches. In the present study, low heterogeneities of meta-analyses were obtained, and according to the funnel plots, no publication bias was observed, which also supported the current results.

Taken together, those results suggest that the reconstruction nail is probably a better treatment option than the hollow screw+plate for the management of patients with femoral shaft and neck fractures. The reconstruction nail has definitive advantages in healing time, union rates, and complications. We consider that the reconstruction nail should be the first choice in most patients.

Nevertheless, the present study had some limitations. First, the indicators and comparisons in this study were limited, which indicated that more indexes need to be analyzed and evaluated in future studies. Second, the included countries were limited, and data in more countries are essential and should be assessed in future studies. Third, the experience of the surgeons was not consistently reported, precluding any analysis of this factor. Fourth, heterogeneity among studies regarding the patients, surgical settings, and devices used may limit the conclusions.

## Conclusion

In conclusion, the current meta-analysis demonstrated the comparison between reconstruction nail and hollow screw+plate. In both clinical efficacy and safety, the reconstruction nail was rendered as an optimal therapy than a hollow screw+plate.

## Data Availability

The datasets used and/or analyzed during the current study are available from the corresponding author on reasonable request.

## Abbreviations

CI: Confidence interval
OR: Odds ratio
